# Computational Methods for Automated Analysis of Malaria Parasite Using Blood Smear Images: Recent Advances

**DOI:** 10.1155/2022/3626726

**Published:** 2022-04-11

**Authors:** Shankar Shambhu, Deepika Koundal, Prasenjit Das, Vinh Truong Hoang, Kiet Tran-Trung, Hamza Turabieh

**Affiliations:** ^1^Chitkara University School of Computer Applications, Chitkara University, Himachal Pradesh, India; ^2^School of Computer Science, University of Petroleum and Energy Studies, Dehradun, India; ^3^Faculty of Computer Science, Ho Chi Minh City Open University, Ho Chi Minh City, Vietnam; ^4^Department of Information Technology, College of Computing and Information Technology, Taif University, P.O. Box 11099, Taif 21944, Saudi Arabia

## Abstract

Malaria comes under one of the dangerous diseases in many countries. It is the primary reason for most of the causalities across the world. It is presently rated as a significant cause of the high mortality rate worldwide compared with other diseases that can be reduced significantly by its earlier detection. Therefore, to facilitate the early detection/diagnosis of malaria to reduce the mortality rate, an automated computational method is required with a high accuracy rate. This study is a solid starting point for researchers who want to look into automated blood smear analysis to detect malaria. In this paper, a comprehensive review of different computer-assisted techniques has been outlined as follows: (i) acquisition of image dataset, (ii) preprocessing, (iii) segmentation of RBC, and (iv) feature extraction and selection, and (v) classification for the detection of malaria parasites using blood smear images. This study will be helpful for: (i) researchers can inspect and improve the existing computational methods for early diagnosis of malaria with a high accuracy rate that may further reduce the interobserver and intra-observer variations; (ii) microbiologists to take the second opinion from the automated computational methods for effective diagnosis of malaria; and (iii) finally, several issues remain addressed, and future work has also been discussed in this work.

## 1. Introduction

Malaria has turned into a major risk to individuals worldwide as one of the main reasons for causalities across the world. It is a curable infectious disease caused by a protozoan parasite that can be life-threatening. As per the latest report of the World Health Organization (WHO), in 2019, 229 million malaria cases were detected worldwide, and causalities were reached to 409000. In 2018, 228 million malaria cases were detected, and causalities were reached 411000 [1].

In 2016 and 2017, about 1.09 million and 0.84 million malaria cases were registered in India, in which most of the malaria cases were *P. falciparum* species affected [2].

Dr. Ronald Ross first discovered malaria transmission in the human body by mosquitoes in 1897 [3]. The main reason for malaria is a protozoan parasite. The plasmodium genus infects the red blood cells (RBC) of the human body, which causes malaria [4]. In general, female *Anopheles* mosquitoes and human beings are the two main hosts infected by the parasite. When female *Anopheles* mosquitoes desire to foster their eggs, they bite and draw blood from the human body. If a parasite infects that person, then that same infected parasite blood is found in the mosquito and that parasite reproduces and develops in the mosquito body. When that infected mosquito bites another person, parasites containing the salivary gland are transferred into that person's blood [5]. After transferring parasites into the human body by the mosquito, malaria parasites grow with very high speed in the liver and RBC of that infected person. Symptoms of malaria appear after one or two weeks. Primary symptoms that appear are headache, vomiting, fever, and chills. If malaria is not treated early and properly, it is very harmful to the human body. It may be a reason for kidney failure, low blood sugar, respiratory distress, enlargement of the spleen, etc. [6]. Malaria can kill a person by destroying their RBC. Malaria during pregnancy is very dangerous, and it is one of the reasons for abortion [7].

There are five different protozoan parasite species, which are the main cause of malaria in the human body. These are *Plasmodium falciparum* (*P. falciparum*), *Plasmodium vivax* (*P. vivax*), *Plasmodium ovale* (*P. ovale*), *Plasmodium malaria* (*P. malaria*), and *Plasmodium knowlesi* (*P. knowlesi*). Among all five species, the first four are the most common species, which occur in the human body. The fifth species is *P. knowlesi* mostly occurs in monkeys that live in South-East Asia forests. But, in past years, some cases of *P. knowlesi* malaria occurred in the human body. The most common species found in the human body is *P. vivax,* but the most dangerous species is *P. falciparum* [8].  Figure 1 shows the images of the different types of malaria found in human peripheral blood smears.

All species of protozoan parasites are morphologically different. At every stage of its lifecycle, each species changes in its size, color, shape, and morphology. These various stages of every species are ring, trophozoite, schizont, and gametocyte, as shown in Figure 2.

The main reason for the high mortality rate is the late detection of malaria. In medical science, for the detection of malaria, microscopic examination is the gold standard. A microbiologist manually counts affected RBC under the microscope to examine the patient's blood sample, which is a very time-consuming and highly tedious process. The accuracy of this process is entirely dependent on microbiologist expertise [10]. Hence, microscopic examination is a prolonged process, and it is the main reason for the late detection of malaria in patients, increasing the high mortality rate. The high malaria mortality rate can be decreased by detecting malaria at an early stage. Therefore, an automated computer-assisted technique is needed, which will help the microbiologists to provide a second opinion for effective and early detection of malaria and reduce the mortality rate.

The pattern of total worldwide malaria patients is illustrated in Figure 3. It represents how malaria patients are increasing worldwide. In 2013, 198 million malaria-affected patients were detected, which was increased to 229 million in 2019 [1]. These very troubling statistics can be reduced by detecting parasites and diagnosis in the early stages, and it would be beneficial when experts are not available.

The paper's contributions are as follows: (i) a comprehensive review has been conducted on the state-of-the-art techniques for malaria diagnosis that have been published in the last decade; (ii) various types of automated computational methods such as preprocessing, segmentation, feature extraction, and classification for diagnosing malaria have been discussed in detail; (iii) additionally, different types of machine learning and deep learning models, as well as their accuracies for malaria parasite detection and diagnosis, have been discussed; (iv) moreover, several types of blood smear image datasets for malaria diagnosis have been identified; and (v) various challenges and issues with the already implemented techniques and scope of future work have also been discussed.

The paper is organized as follows: (i) Section 2 summarizes the state-of-the-art techniques for malaria diagnosis; (ii) Section 3 explains automated computational methods for diagnosing malaria in detail; (iii) Section 4 presents the discussion with research gaps; and (iv) Section 5 concludes the paper with future scope.

## 2. State-of-the-Art Techniques for Malaria Diagnosis

Malaria is a disease in which symptoms appear after 7 to 15 days. Primary symptoms are headache, vomiting, fever, pain, chills, etc. These symptoms could be an indication of malaria, although many diseases have the same symptoms. Hence, some techniques are needed that can diagnose malaria correctly. For malaria diagnosis, different techniques have been developed such as microscopy blood smear examination, cytometry, rapid diagnostic test (RDT), polymerase chain reaction, and fluorescent microscopy. Still, for diagnosing malaria, the primarily used techniques are (a) microscopic thick and thin blood smears examination and (b) rapid diagnosis test in medical science [11].

### 2.1. Microscopic Thick and Thin Blood Smears Examination

In this, a laboratory examination is performed in which a clinician divides the blood sample into two parts on the slide. One is called a thick blood smear, and another is a thin blood smear. After that, a clinician manually counts the affected RBC under the microscope. A thick blood smear helps clinicians detect the presence of malaria parasites, and a thin blood smear helps identify the species of the parasites causing malaria. All the steps for malaria detection using microscopic blood smears examination are shown in Figure 4.

Advantages of the microscopic technique are as follows: (i) a clinician can distinguish the different stages of malaria species at a very low cost using microscopic method and (ii) microscopy technique for malaria detection is more effective as compared to rapid diagnostic tests as it can count affected RBC very efficiently. Apart from the advantages of microscopic techniques for malaria detection, some challenges are also there. Microscopic thick and thin blood smears examinations technique accuracy depends on microbiologist experience. To detect and diagnose malaria through a microscope, a microbiologist may have to count malaria-affected RBC manually, which is a highly tedious and time-consuming task [10]. It is found in multiple studies that manual counting of affected cells using a microscope is not an authentic technique when it is done by a nonexperienced microbiologist [13]. Instead of this, to confirm a blood smear slide is malaria-affected or not, a microbiologist needs significant time. But, it is a tough task for a microbiologist to examine each slide because a microbiologist has to study multiple blood smear images under the microscope. Moreover, this technique takes time to examine blood smear slides.

### 2.2. Rapid Diagnosis Test (RDT)

Rapid diagnosis test or antigen test is a small kit used to detect antigens derived from malaria parasites. To identify malaria, a drop of blood is inserted into the kit from the given hole, and internally, this device performs the tests and provides the result in minimum time. RDT kit functioning is shown in Figure 5.

Advantages of the RDT kit are as follows: (i) it is significantly faster than manual cell counting techniques, and it gives instant results; (ii) for the use of the RDT kit, no expertise is required; and (iii) it is beneficial in endemic regions. Instead of the advantages of the RDT kit for malaria detection, some challenges are also there. As per the analysis of different studies, the results of this technique are less accurate, and any wrong result can affect the patient's treatment [14]. Another main challenge of the RDT kit is detecting whether a patient is malaria-affected or not. It cannot detect malaria species.

Hence, after studying different techniques of malaria diagnoses and their advantages and challenges, researchers observed that a computer-assisted malaria detection technique would be required. A computer-assisted malaria detection technique increases the performance of existing techniques by avoiding its limitations in terms of accuracy, instant results, dependency, and requirement of the expert microbiologist.

## 3. Automated Computational Methods for Diagnosis of Malaria

In medical science, the computer plays a very crucial role. Different automated computational methods are used for the diagnosis of multiple diseases. Ultrasound images, magnetic resonance imaging, X-ray images, and computed tomography images are used to diagnose different diseases of human anatomy using computerized imaging techniques. The computer-assisted diagnosis technique for malaria is based on the microscopic technique, which is performed by computer with the help of machine learning algorithms and computer vision techniques. This is the technique in which digital thin and thick blood smear images are used for the detection of malaria parasites automatically. Different steps of automated diagnosis of malaria are image acquisition, preprocessing, red blood cell detection and segmentation, feature extraction, and selection and classification (parasite identification and labeling). The stepwise process of automated computational methods for malaria parasite diagnosis is shown in Figure 6. In this section, a deep survey has been performed on each technique used for automated detection of malaria using blood smear images.

### 3.1. Acquisition of Image Dataset

Digital images of blood smear samples are required to detect malaria in a patient using computer vision image processing and machine learning techniques. Each patient's blood smear sample is distributed into two parts: thick and thin blood smear images. Most computer-assisted detection studies use thin blood smear digital images, and very few researchers have worked on thick digital blood smear images [16].

Figure 7 shows the images of thick and thin blood smears. A thick blood smear is a drop of blood that assists in detecting the presence of parasites, and a thin blood smear is a layer of blood that is spread on a glass slide and assists in identifying the species of the parasite causing the infection. Different sources collect digital blood smear images, and this process is called the image acquisition technique. Categorization of different image acquisition techniques used on blood smear images for malaria parasite detection is shown in Table 1.

After analyzing the different image acquisition techniques in Table 1, we observed that there are various image acquisition techniques available. Still, the light microscopy technique is the most widely used and preferred because it has a high magnification factor, and it is beneficial for viewing the surface details of a blood smear.

Furthermore, Table 2 lists the different datasets of light microscopy techniques used by various researchers.

### 3.2. Preprocessing

Preprocessing is a technique used to remove the unwanted noise and produce high contrast digital blood smear images for the next step. When different resources take blood smear images, the images are corrupted by noise, and thus, visualization of the images is not good. Due to this problem, further steps of segmentation and classification are challenging to implement, and it produces poor results. Hence, certain preprocessing techniques have been used to remove that unwanted noise from images. Preprocessing techniques remove the noise from the image for better visualization, which is very useful for further analysis [46]. As shown in Table 3, researchers used multiple preprocessing techniques such as median filter, mean filter, low-pass filter, morphological filter, partial contrast stretching, local histogram equalization, Laplacian filter, SUSAN filter, geometric mean filter, Gaussian filters, and Wiener filter for enhancing the contrast and remove the unwanted noise of digital images. May et al. have given an approach in which the median filter technique for removing the impulse noise from digital images and for removing additive noise has been used [4]. The Gaussian filter is used by Arco et al. to enhance the quality of the images affected by Gaussian noise. The geometric mean filter is also used by Das et al. for preserving the edges and removing Gaussian noise from the digital microscopic image [66]. Laplacian filter is used by Savkare et al. for smoothening and enhancing edges of malaria parasite images [29]. To preserve the structure of an image, Susan's filter is suggested by [41]. To remove the intensity of high frequency from a digital image, a low pass filter has been suggested by [55]. The histogram matching technique is used by Abbas et al. to normalize the intensity value of digital image pixels [67]. The categorization of preprocessing techniques to enhance the quality of digital blood smear images is shown in Table 3.

Table 4 displays the image preprocessing approaches used by various researchers for better visualization of thin and thick blood smear images with their properties.

### 3.3. Red Blood Cell Detection and Segmentation

Segmentation is the process in which digital images are disjoint into nonoverlapping regions. Each disjoint image typically corresponds to other parts of an image object. Once each digital image object is isolated, each object can be easily measured and classified. In the literature, different segmentation techniques have been applied on digital blood smear images to detect ROI (region of interest).

Das et al. have developed an automated system for classifying malaria at different stages. The researcher used the watershed segmentation technique in their research work for the segmentation of thin blood smear digital images. This technique provided better results for detecting erythrocytes from the whole blood smear image [66]. Further, a watershed algorithm is suggested by Savkare et al. to find overlapped cells on connected components [29]. Soni et al. used the granulometry technique [41]. Makkapati and Rao have developed a technique to segment RBC and parasites using HSV (hue, saturation, and value) color space. This technique segmented the RBC and parasites from the blood smear image based on hue range and optimal saturation thresholds [69]. Mandal et al. introduced a normalized cut method for microscopic blood smear images segmentation.

The segmentation algorithm has been used on different color spaces to find the optimal performance of digital blood smear images [70]. The result of the normalized cut segmentation algorithm is good in HSV color space. Nasir et al. have presented a segmentation-based approach using a K-means clustering algorithm for the segmentation of malaria parasite on 100 digital blood smear images dataset [71]. Bhatia also proposed a K-means clustering technique using genetic methods [72]. Panchbhai et al. have reported the RGB color space model and Otsu algorithm for RBC and parasite segmentation from 20 thin blood smear images [73]. For microscopic blood cells, digital images segmentation, the K-means clustering technique, and global threshold techniques are suggested by Savkare and Narote [74]. In this, 78 microscopic blood cell digital images are used for segmentation. Khan et al. also used the K-means clustering for the segmentation of 118 blood smear images to identify malaria parasite tissues [75]. Acharya et al. introduced a new computer-assisted detection technique for segmenting blood smear images and determining the acute myeloid leukemia stage (AML). This work's approach is divided into many stages. A unique algorithm is being developed to accurately segment blood smear images in order to identify AML and its variants. The classification accuracy of the model was 99.48% on 500 test images [76].

To detect the exact radius of RBC, the circle hough transformation method was introduced by Ma et al. [77]. Otsu thresholding clustering-based method is presented by Makkapati et al. to get the image mask of binary image [78].

Deep learning techniques are also beneficial in image segmentation. Researchers for image segmentation have proposed many deep learning techniques. For image segmentation, a fully convolutional neural network-based deep learning technique has been proposed by Long et al. [79] and Wang et al. [80]. A completely CNN encoder and decoder deep learning segmentation technique (SegNet) has been used by Badriinarayanan et al. [81]. Ronneberger et al. proposed the U-Net to segment biomedical microscopic images [82]. Dai et al. created a multifunction network, for instance segmentation that includes three networks for separating instances, computing masks, and labeling objects. These networks must share their convolutional characteristics and form a cascaded structure [83]. Visin et al. have used ReSeg, an RNN-based deep learning approach for semantic segmentation of the images. This approach is primarily based on the image classification model ResNet [84].

Segmentation techniques on blood smear images used in different studies are summarized in Table 5. After analyzing various segmentation techniques, it was found that for the segmentation of malaria parasites and RBC, most researchers used Watershed, Marker-controlled watershed, and Edge detection algorithm, and deep learning techniques at the segmentation phase. For the segmentation of overlapping cells, watershed algorithm results are best [28].

### 3.4. Feature Extraction and Selection

Feature extraction after segmentation is a prerequirement for feature selection and classification. The objective of feature extraction is to recognize and characterize an object whose dimensions are very nearest or similar for objects in the same class and different for objects from a different class. It reduces the computational complexity of the other processes and provides accurate and reliable recognition to unknown, unrecognized data.

To develop a good classification model, a good feature selection method plays a very important role. Classification model processing time and results of classification model depend on selection and type of the number of selected features or attributes. In the literature, several researchers have developed and used different feature selection methods.

To extract the features of haralick textures, mean, entropy, roughness, homogeneity, and standard deviation, Das et al. suggested gray-level co-occurrence matrix [66]. To extract the intensity-based features, Chayadevi and Raju used a color channel intensity algorithm [96]. Rajaraman et al. have given a pretrained model for the feature extraction and the detection of malaria parasites [101]. In this, a pretrained convolutional neural network including AlexNet, VGG-16, Xception, ResNet-50, and DenseNet-121 are used for extracting features from infected and uninfected 27558 cell images. The developed model for feature extraction and malaria parasite detection took more than 24 hours for training and produced 95.9% accuracy for malaria parasite detection in thin blood smear images. To identify the texture features from a blood smear image to detect malaria parasites, Chavan and Sutkar used a histogram-based feature extraction method [102]. The color histogram feature extraction technique is used by [43] for identifying infected erythrocytes from blood smear images. Reference [103] extracted features of RBC size and shape, RBC texture, and parasite shape from the thin blood smear images, and used these features to classify malaria parasite species. For extracting the features from digital microscopic images based on morphological, [43] used a granulometry algorithm.

Various features of extraction and selection techniques implemented by various researchers for malaria blood smear images are shown in Table 6. As evident from Table 6, it is found that researchers used different feature extraction techniques based on their goals. Mostly used feature extraction techniques were color features and texture features. However, some authors recommended morphological feature technique for features extraction from malaria blood smear images [51, 108].

### 3.5. Parasite Identification and Labelling (Classification)

Classification is a technique to identify a pattern that belongs to which class. In this literature, different authors developed different classification techniques to identify a patient, whether he or she is malaria-affected or not. So, there are two classes to detect whether the patient is affected by malaria or not.

Vijayalakshmi and Kanna have introduced a deep learning approach to classify infected and noninfected falciparum malaria. The presented technique was achieved by the visual geometry group (VGG) network and SVM. In this, 1530 malaria digital corpus images have been used for training and testing the model. In this, the transfer learning approach to train the model is used in which we trained the top layer of the model and freeze the rest out of the layers approach applied. For the classification of infected or noninfected falciparum malaria, the given model obtained 93.13% accuracy [8].

For the classification of malaria-infected stages from thin blood smear images, Das et al. used five different classifiers to classify the malaria-infected stages. These five classifiers are Naive Bayes, Logistic regression, Radial Basis Functions (RBF) neural network, Multilayer perceptron neural network, and classification and regression tree. In this, 888 erythrocytes infected and noninfected image dataset is used. Out of this, 592 labeled images are used to train the classifiers and the remaining are used for testing the classifiers. The experimental results show that among all five classifiers, the multilayer perceptron network has provided better results than the other four classifiers on the 750 images dataset [66].

Seman et al. developed a multilayer perceptron network (MLP) to classify different malaria parasite species from thin blood smear images. This work classified three different species from malaria parasites: *P. falciparum, P. malariae, and P. vivax* [103]. The authors used the backpropagation algorithm of the MLP network for training and compared the results of the MLP network with Levenberg–Marquardt and Bayesian rule algorithms. MLP network has produced better results as compared to the other two algorithms.

Otsu thresholding method is used by Malihi et al. for the classification of four species of malaria parasites in blood smear images. This technique has provided better results in comparison with other techniques. In this, 363 blood smear images are used and obtained 91% accuracy [43].

Further, Anggraini et al. have classified the different stages of malaria parasites using a Bayesian classifier on 110 thin blood smear images and obtained 93.3% accuracy [112]. Minimum distance classifier technique has been given by Ghate et al. for detecting the presence of malaria parasites using 80 blood smear images and got 83.75% accuracy [39]. Savkare and Narote presented Otsu thresholding, watershed transform, and SVM binary classifier to classify normal and parasite-infected cells [113]. Das et al. have presented the Bayesian approach for automated screening of malaria parasite from microscopic images [51].

Kareem et al. have developed an automated technique for detecting malaria parasites in thin blood smear images. In this, a dataset of more than 200 images is used. Two methods of classification for parasites are used. The first one is based on relative size and morphology, and the second is based on intensity variation. The final results of the developed model have shown an accuracy rate of 87% [36].

Prasad et al. have presented a decision support system approach to classify the infected and noninfected malaria parasites in thin blood smear images. In this, 200 thin blood smear images have been used, and 96% accuracy has been obtained [114]. Rosado et al. have developed a supervised classification technique to detect malaria parasites in blood smears. In this, machine learning (ML) classification 10-fold cross-validation for WBC (white blood cell) and P. falciparum trophozoites detection has been performed and got 91.8% accuracy [85].

Mohammed and Abdelrahman have given a technique for detecting and classifying malaria from 160 thin blood smear images taken from the Centre for Disease Control and Prevention (CDC). To extract the RBC from blood smear images, researchers used morphological processing. This technique found the parasites and overlapped cells in the image. Based on the number of RBCs in each image, RBC is classified into two classes: infected and noninfected cells. After that, a normalized cross-correlation algorithm was employed to classify the affected blood smear parasite into four different malaria species. The given method has produced 95% accuracy for detection [23]. Saiprasath et al. evaluated seven different machine learning algorithms on the same malaria image dataset and concluded that Random Forest outperforms every other algorithm, closely followed by the Ada Boost algorithm [115].

Bibin et al. have given an automated technique to detect malaria parasites in peripheral blood smear images. The given binary classifier is based on deep learning, which used 1978 images to train and test the technique and achieved 96.21% accuracy [106]. Simon et al. suggested a CNN-RNN model for malaria detection. Compared with the CNN-LSTM and CNN-GRU models, the proposed model generated the best results [116]. Dev et al. suggested a hierarchical convolutional network and produced better results than prior studies [117].

Dave et al. used adaptive thresholding, erosion, and dilation operations to diagnose malaria from 117 blood smear microscopic digital images and got 89.88% accuracy [34]. Oliveira et al. have suggested the face detection algorithm to identify Plasmodium parasites from blood samples. In this, a dataset of 1332 blood sample images has been taken and shown 91% accuracy [118].

Mohanty et al. have presented the autoencoder (AE) neural network unsupervised technique to identify malaria in blood smear images. In this, the AE technique has been compared with the SOM technique. The AE technique obtained 87.5% accuracy compared to the 79% accuracy of the SOM technique. 1182 blood smear images have been used to perform experiments [119]. Morales-Lopez et al. suggested the SVM technique for classification problems [120].  Table 7 has listed different types of classification techniques used for the identification of malaria parasites.

After the analysis of Table 7 and literature of malaria parasite classification techniques, it is found that various classification techniques that researchers commonly implement are CNN, SVM, and TL-VGG classifiers.

## 4. Discussion

In the last decade, a lot of experiments have been done in the area of automated detection of malaria to reach the current state-of-the-art. In this study, different computational methods implemented on various stages of computer-assisted techniques for detecting malaria parasites using blood smear images have been examined. Image acquisition is the first and very important step for automatic detection of the malaria parasite. The present study shows various techniques for acquiring digital blood smear images, but the light microscopy technique is the most widely used and liked technique by researchers. There is a number of computational methods out of which preprocessing is the first step in image analysis.

Preprocessing is one of the crucial stages implemented on acquired digital blood smear images. It plays a crucial role in detecting infected RBC by removing the unwanted noise and producing high contrast digital blood smear images without demolishing the image features. As per the current study, median/mean filter, morphological filter, Laplacian filter, Susan filter, and Gaussian low-pass filter are mostly used techniques by researchers to remove unwanted noise and increase the contrast of the images. Segmentation is the next stage after the preprocessing, which is used to segment the RBC to detect malaria parasites using blood smear images to facilitate the classification process. As per the study of literature, mostly used segmentation techniques by researchers are as follows: (i) Otsu thresholding for segmentation of parasite RBC; (ii) Marker-controlled watershed and Edge detection algorithm is used at the segmentation phase; and (iii) for the segmentation of overlapping cells, the watershed algorithm has been widely used.

After segmentation, blood smear images have been classified to diagnose malaria-infected or not infected by feature extraction and selection techniques. As per the study, Color features, Texture features, and Morphological features have been mostly used feature extraction techniques for early diagnosis of malaria from blood smear images. From the literature, it has been observed that the maximum accuracy of 95.03% has been achieved by CNN based deep learning model in comparison with the VGG-SVM model [8, 101, 126].

A thorough review of the literature on automated analysis of malaria parasite using blood smear images yielded the following challenges and future directions:

The accuracy of an automatic image classification model depends upon multiple aspects such as analysis of the digital blood smear image depend on the staining method, magnification factor of an image, condition of nearest environment where the digital image has been collected like the background of the image, light in the room, and most important quality and position of the camera. Therefore, a standard digital blood smear dataset is necessary to test and validate the model to obtain efficient and reliable results.

Many researchers have performed their experiments and published their articles in the same area. Moreover, an automated computational-based computer vision method, which should be efficient and effective for automated detection of the malaria parasite from blood smear images, needs to be improvised according to the requirement of the community.

The community requires (i) standard image dataset because researchers' datasets are mostly unstandardized. The digital blood smear dataset depends on the characteristics and quality of the microscope as all digital images of blood smears are taken by a digital camera attached to a microscope. So, a well-standardized dataset is most important for a machine learning algorithm for automated detection of malaria. (ii) In the literature, developed methods can recognize only one type of malaria parasite [8]. But, the patient may be affected by more than one parasites species. Hence, there is a need for such a model that can recognize different types of malaria parasites. (iii) To classify malaria parasites from blood smear images, authors trained the machines with different models and techniques. The training model is taking a long time to learn [66]. Hence, there is a necessity to reduce the training time to train the classification models. (iv) In literature, developed models by different researchers analyze the blood smear digital images that are taken from a camera that is attached with a microscope [4, 8]. Hence, there is a demand for a model to analyze thin blood smears images acquired exclusively with smart phones [43]. (v) A technique that different authors use to diagnose malaria is invasive, in which an injection syringe takes a blood sample. Therefore, there is a requirement for a noninvasive technique that can be used to detect malaria [128]. (vi) After the analysis of Table 7, it has been found that all the existing state-of-the-art techniques used to detect malaria from microscopic blood smear images are not very accurate. Each technique has some limitations and challenges. Therefore, there is a necessity for an automatic technique that can improve the accuracy for the detection of malaria parasites and it will also help in early detection of malaria and reduce the mortality rate in future.

## 5. Conclusion

This study is a solid starting point for researchers who want to look into automated blood smear analysis to detect malaria. This study reviews and discusses computer vision and image analysis works that target the automated detection of malaria on blood smear images. In this paper, we have discussed the present facts of necessary components of computer-assisted technique: (i) acquisition of image dataset, (ii) preprocessing, (iii) segmentation of RBC, (iv) feature extraction and selection, and (v) classification, which have been used to diagnose malaria parasite from blood smear images suggested by various researchers. Digital blood smear images taken from a microscope may affect how and which malaria parasites are detected. After analyzing segmentation and classification state of the art techniques, it has been observed that future computer-assisted techniques should be based on standard datasets and magnification factors to detect malaria parasites. The complexity of different classifiers of machine learning that are based on deep learning increases as the number of layers increases. To achieve efficient and reliable results, a large dataset is required for training and testing. With the help of computational methods such as data augmentation and deep learning methods, the computer-assisted method can obtain better results.

However, some state-of-the-art techniques are presented in the literature, but still, there is a huge scope of future work, which may help the microbiologists in the detection and diagnosis of the malaria parasite at an earlier stage to reduce the mortality rate such as (i) different computational methods that are used to collect blood smear images physically can be studied more to enhance the segmentation results to detect infected RBC very effectively. Hence, an efficient computational method of infected RBC segmentation can be developed. (ii) Various feature extraction methods such as color features, texture features, and morphological features [51, 106, 108] can be analyzed more, which will be very helpful for the development of an efficient automated computer-assisted system to detect infected malaria RBC using blood smear images. (iii) To classify malaria blood smear images, mostly implemented techniques are SVM, K-means, and VGG classifiers. Still, there is a vast scope to implement customize CNN algorithms to detect infected malaria RBC with high accuracy. If the CNN model is implemented on blood smear images at a minimum magnification factor for classification, it may decrease the cost and time complexity of the system.

In the field of malaria detection from blood smear images, the contribution of many research publications is noteworthy. However, this study has tried to present opinions to the microbiologists and technical community. It will be very helpful for them to generate an effective and efficient computer-assisted technique for malaria detection at an early stage. [129, 130].

## Figures and Tables

**Figure 1:** Different types of malaria peripheral blood smear images (a) P. falciparum (b) P. vivax (c) P. ovale (d) P. malaria [9].

**Figure 2:** Different stages of malaria parasite species.

**Figure 3:** Worldwide year-wise prevalence count of malaria patients.

**Figure 4:** Microscopic thick and thin blood smears examination [12].

**Figure 5:** Rapid diagnosis testing (RDT) kit [15].

**Figure 6:** Computational methods for automated diagnosis system for malaria.

**Figure 7:** Malaria infected thin (left) and thick (right) blood smear image.

**Table 1:** Categorization of image acquisition techniques used on blood smear images for malaria parasite detection.

References	Light microscopy	Binocular microscopy	Fluorescent microscopy	Polarized microscopy	Multispectral and multimodal microscopy	Image-based cytometer	Scanning electron microscopy
[17]	✓						
[18]			✓				
[19]	✓						
[20]	✓						
[21]	✓						
[22]			✓				
[23]	✓						
[24]						✓	
[25]	✓						
[26]	✓						
[27]		✓					
[28]	✓						
[29]	✓						
[30]				✓			
[31]					✓		
[32]	✓						
[33]	✓						
[34]			✓				
[35]							✓
[36]	✓						
[37]					✓		
[38]		✓					
[39]	✓						
[40]	✓						
[41]		✓					
[42]			✓				

**Table 2:** Light microscopy datasets used by different researchers.

Reference	No. of images in dataset	Remarks
[43]	300 images	Used KNN classifier on light microscopic images, got 91% accuracy.
[33]	21 images	Light microscopic images of 1296 × 1024 resolution captured by an axiocam high-resolution color camera were used.
[44]	—	—
[29]	68 images	Light microscopic images of different magnification have been used.
[25]	300 images	Used KNN classifier and got 90.17% accuracy to detect malaria parasite species.
[26]	27578 images	27578 single cell light microscopy images were used, and a new 16-layer CNN model was proposed to identify malaria-infected or infected images.
[23]	160 images	Achieve 95% accuracy for the detection of malaria.
[45]	—	Used Giemsa-stained blood smear images were taken by a camera attached with a microscope on 1000x magnification, and the proposed model got 77.78% accuracy.
[19]	27558 images	Implement novel stacked convolutional neural network technique for parasite detection.

—Not reported by the original paper.

**Table 3:** Categorization of preprocessing techniques used on blood smear images.

References	MMF	LPF	MF	PCS	LHE	LF	SF	GMF	GF	WF
[47]	✓									
[48]										✓
[49]							✓			
[50]	✓		✓							
[29]	✓					✓				
[51]								✓		
[52]						✓				
[53]				✓						
[54]					✓					
[55]		✓								
[21]			✓							
[27]	✓									
[20]	✓									
[56]									✓	
[38]							✓			
[57]					✓					
[43]	✓									
[58]	✓									
[59]			✓							
[60]			✓							
[61]					✓					
[62]					✓				✓	
[63]	✓									
[64]			✓							
[24]	✓									
[65]			✓							

MMF—median/mean filter; LPF—low pass filter; MF—morphological filter; PCS—partial contrast stretching; LHE—local histogram equalization; LF—Laplacian filter; SF—SUSAN filter; GMF—geometric mean filter; GF—Gaussian filters; WF—Wiener filter.

**Table 4:** Thin and thick blood smear based preprocessing techniques used for better visualization.

Type of blood smear	Problems	Reference	Preprocessing technique used	Remarks	Limitations/challenges
Thin blood smear image	Noisy blood smear image	[20, 27]	Median/Mean filter	Used to remove noise from blood smear images without affecting the edges.	The presence of impulse noise cannot be eliminated. It impacts the average rating of all pixels in the surrounding area.
		[48]	Wiener filter	Used to enhance the quality of blurred images.	The power spectra are difficult to estimate.
		[38, 49]	SUSAN filter	Helpful for finding the edges corners and for noise removal.	The brightness similarity metric is significantly affected by the threshold.
		[55]	Gaussian low-pass filter	For removing Gaussian noise in blood smear images, Gaussian low-pass filter was used.	Take too much time.
		[51]	Geometric mean filter	Useable for maintaining edges while removing Gaussian noise.	A negative observation will result in an imaginary geometric mean value regardless of the other observations' quantity.
		[21, 50, 59]	Morphological filtering	Helpful for deleting unwanted objects, filling small holes, and splitting images.	When using morphological operators, it is necessary to consider the concepts of infimum and supremum.
	Low contrast blood smear image	[53]	Partial contrast stretching method	Used to increase the contrast of the blood smear image.	—
		[29, 52]	Laplacian filter	Helpful for detection and improving the edges of the blood smear image.	The detection of edges and their directions increases the noise in the image, reducing the edge magnitude.
		[54, 57]	Local histogram equalization	Used to increase the resolution of blood smear images.	It is an indiscriminate technique.
	Unequal illumination	[62]	Low-pass filter	For removing excessive frequency components from blood smear images.	—
	Variations in cell staining	[20]	Gray world color normalization	Used for equality of color in blood smear images.	Poorly constructed normalization software might result in a reduction in the entire image quality.
Thick blood smear image	Noisy blood smear image	[68]	Gaussian low-pass filter		Take too much time.
			Laplacian filter		The detection of edges and their directions increases the noise in the image, reducing the edge magnitude
			Median filter		
			Local histogram equalization		
			Contrast enhancement method		

—Not reported by the original paper.

**Table 5:** Summary of segmentation techniques used on digital blood smear images.

References	Segmentation techniques used	Remarks	Limitations/Challenges
[4, 29, 43, 85–88]	Otsu thresholding	Classification of pixels by using a calculating optimum threshold value.	In the case of global distribution, this algorithm fails.
[23, 26, 31, 79–81]	Histogram thresholding	The quality of segmentation depends on the threshold value.	Deciding the threshold value is a crucial task.
[25, 53, 71, 75]	K-means clustering	Unsupervised segmentation technique used to obtain the same feature regions.	The value of the cluster, i.e., K, must be defined.
[28, 29, 89]	Watershed algorithm	Used for continuous boundary regions extraction. Gives good results on overlapping cells.	The calculation of gradients is complex.
[20, 38, 51, 59, 66, 88]	Marker-controlled watershed	Used to separate overlapped cells.	Does not work on extremely overlapped cells.
[23, 33, 43, 62, 90]	Morphological operation	Mathematical operations are used to separate RBC based on size, texture, boundaries, gradient, circular shape, etc.	High time complexity.
[28, 32, 91–93]	Edge detection algorithm	Excellent results on high contrast and sharp edge blood smear images.	It is a time-consuming process if there are many edges.
[94, 95]	Rule-based segmentation	Required understanding of color, shape, and size of RBC.	RBC's color, size, and shape understanding are required.
[96–98]	Fuzzy rule-based segmentation	Rules need to be designed for segmentation, which is a complex task.	Designing rules is a complex task.
[21, 77, 99, 100]	Hough transform	Used to segment accurate radius and shape of cells.	Computationally expensive in case of a large number of parameters.

**Table 6:** Different techniques used for the extraction of features and selection from malaria blood smear images.

References	Color features						Texture feature									Morphological feature		
	RGB	HSV	YCbCr	Lab	Intensity	CCM	Haralick	GLRLM	GLCM	LBP	Fractal	WT	GT	Entropy	SIFT	Shape	Moments	Area
[24]	✓																	
[104]	✓															✓		
[105]					✓											✓		
[106]		✓					✓		✓	✓								
[96]	✓	✓																
[70]	✓		✓															
[107]																✓	✓	
[108]	✓											✓	✓				✓	
[109]														✓			✓	
[51]								✓		✓				✓		✓	✓	
[100]							✓	✓								✓	✓	
[25]				✓														
[110]						✓		✓		✓	✓							
[111]															✓			
[43]	✓												✓					✓
[38]																		✓
[66]									✓									
[102]																		
[65]					✓				✓									
[21]														✓			✓	
[20]	✓																	
[31]	✓				✓													

RGB—red green blue; HSV—hue, saturation, and value; CCM—color co-occurrence matrix; GLRLM—Gray-level run length matrices; GLCM—gray-level co-occurrence matrix; LBP—local binary pattern; WT—wavelet transform; GT—gradient texture.

**Table 7:** Different classification techniques used for the identification of malaria parasites.

Reference	Technique used	Dataset	Accuracy (%)	Limitations/challenges
[103]	Multilayer perceptron network for classification of malaria species.	562 malaria images	89.90	Computation cost is very high.
[113]	Otsu thresholding, watershed transform, and SVM binary classifier for classification of normal and parasite-infected cells.	15 malaria images	93.12	Species detection of malaria is not done. Not suitable for large datasets.
[121]	Comprehensive CAD techniques with 10-fold cross-validation.	1182 malaria images	89.10	Training and testing time is very high for large datasets.
[93]	Suggested SVM technique to find the different stages of infected malaria parasite	530 malaria images	86	Feature scaling is required.
[73]	Used RGB color space model and Otsu algorithm for RBC and parasite segmentation from thin blood smear images.	20 malaria images	92	The unpredictability and imperfections in microscope pictures make precise detection difficult.
[114]	The decision support system for the classification of an infected and noninfected parasite of malaria.	200 malaria images	96	FP rate is 20% and used only thin blood smear images.
[122]	Used minimum distance classifier to detect malaria parasites in blood smear images.	80 malaria images	83.75	Dataset size is very small.
[43]	Used SVM, NM, KNN, 1-NN, and Fisher classifiers to classify different malaria species.	363 malaria images	91	Using a hybrid approach, results can be improved.
[51]	Used Bayesian algorithm for detection of the malaria parasite.	888 malaria images	84	Detect only 1 stage of malaria.
[123]	An artificial neural network has been used to identify the different malaria species from malaria parasites' blood smear images.	200 malaria images	79.7	Performance can be improved by extracting more features.
[96]	Used the neural network method to identify infected RBC from blood smear images.	476 malaria images	94.45	Results can be improved by training the model on a large dataset.
[75]	K-means clustering has been used for the segmentation of malaria parasites cells.	118 malaria images	95	Other types of parasites are not detectable with this technique.
[74]	For the segmentation of RBC, the K-means clustering technique and global threshold technique have been used.	78 malaria images	95.5	Dataset size is minimal.
[66]	For the classification of gametocyte stage and ring stage of malaria species, multilayer perceptron network and 4 other classifiers have been used.	750 malaria images	96.73	By increasing training size, more accurate results can be achieved.
[124]	Used artificial neural network (ANN) for the detection of malaria parasite using morphological features.	7 malaria images	73.57	Achieve better results by increasing dataset size and using 2 or more classifiers.
[85]	Used SVM classifier for WBC and *P. falciparum* trophozoites detection.	1843 malaria images	91.8	Implemented only with the mobile-based framework.
[125]	Used image processing and artificial intelligence techniques and face detection algorithm to identify plasmodium parasites from blood samples.	1332 malaria images	91	Detected only 1 malaria parasite, and more algorithms can explore to achieve better accuracy.
[106]	Malaria parasite detection using a deep belief network.	1978 malaria images	96.21	The technique was not implemented on a dataset acquired from a mobile phone.
[119]	Used autoencoder neural network technique to identify malaria in blood smear images.	1182 malaria images	87.5	The segmentation technique can be improved.
[101]	Used 6 pretrained CNN for feature extraction and subsequent training for malaria parasite detection in thin blood smear images. This model took more than 24 hours for training.	27558 malaria images	95.9	The model took more than 24 hours for training.
[8]	Used transfer learning approach based on VGG-SVM model to classify infected and noninfected falciparum malaria parasite.	1530 malaria images	93.13	A trained model can recognize only 1 falciparum malaria parasite.
[126]	Used CNN based deep learning model (VGGNet-16 architecture) for malaria parasite detection.	27558 malaria images	95.03	Results can be improved by implementing the VGG-19 architecture.
[127]	Used custom CNN that consists of three fully connected convolutional layers.	17460 malaria images	95	A model can test on more computing power systems for better results.

## Data Availability

Dataset is available at https://www.kaggle.com/iarunava/cell-images-for-detecting-malaria.
